RETRACTED

# Analysis of Expression of Inflammatory Factors and T Cell Lymphocyte in Patients with Orthopedic Trauma after Infection and Risk Factors

**DOI:** 10.1155/2022/5387005

**Published:** 2022-09-28

**Authors:** Yuan Lin, Xiao Lei Chen, Tong'en Zhang

**Affiliations:** Department of Joint Surgery and Sports Medicine, Zhongshan Hospital Xiamen University, Xiamen 361004, China

## Abstract

Since most orthopedic patients' wounds are open in clinical practice, postoperative wound infection and other conditions are prone to occur, which pose varying degrees of threat to patients' prognosis and life and health. In this paper, a retrospective study is conducted on orthopedic trauma patients in our hospital from January 2020 to January 2022, including 98 patients with postoperative infection and 98 patients without infection, to detect and compare the levels of inflammatory factors and the level of T cell lymphatic group index difference. The ROC curve is drawn to analyze the diagnostic efficacy of postoperative infection indicators for patients with orthopedic trauma. The differences in baseline data between the two groups are compared. Multivariate Logistic regression analysis is performed on infection status. The experimental results show that the IL-6, IL-2, and CRP of the infection group of patients are significantly higher than uninfected group, and the CD3, CD4, and CD8 are significantly lower than uninfected group, which means that patients with infection after orthopedic trauma are in a disordered state of immune cytokines and function. Therefore, postoperative infection can be effectively assessed by early combined detection of the above indicators. In addition, the analysis of other clinical data showed that the operation time, the number of underlying diseases, and the surgical method are also risk factors for postoperative infection.

## 1. Introduction

There are many factors causing orthopedic trauma. The increase of traffic accidents and accidental injuries has significantly increased the number of orthopedic trauma patients in hospitals [1]. The wounds of orthopedic trauma patients are usually open, so they are prone to complications such as wound infection. Wound infection of patients will not only have a certain impact on patients but also even threaten their lives [2]. The main reason for infection in open wounds is that the skin at the fracture site is damaged, which leads to the contact between the surrounding tissues at the fracture site and the outside world, and the continuous invasion of pathogenic microorganisms, leading to the occurrence of related infection after surgery [3]. Incidence of postoperative infection patients in a clinical study showed that wound healing time, hospitalization time, and the incidence of infection related complications are significantly higher than noninfectious patients; wound healing and longer duration of hospitalization not only bring physical discomfort to patients but also increase the hospitalization time and hospitalization cost, causing certain economic burden to patients [4, 5]. Therefore, reducing the postoperative infection rate can not only effectively accelerate wound healing but also reduce the length of hospital stay and medical expenses [6]. How to evaluate the postoperative infection and its related risk factors is still a hot topic for clinical doctors and patients in the common.

RETRACTED

This paper selects patients with fracture wound in parallel operation to analyze its inflammatory factor and the expression of T cell lymphatic group differences and analyze the risk factors for postoperative infection. This paper provides theoretical guidance for reducing the postoperative infection rate, evaluating the occurrence of infection in time, and taking corresponding measures to reduce the inflammatory response.

The rest of this paper is organized as follows: Section 2 discusses related work, followed by the clinical information and the proposed treatment methods designed in Section 3.  Section 4 shows the experimental results and analysis, and Section 5 summarizes the views of the thesis and points out the future research directions.

## 2. Related Work

In recent years, with the continuous development of modern society and the popularization of various means of transportation, the number of orthopedic trauma patients has increased year by year due to the gradual increase of traffic accidents. In addition, accidental injuries can also cause orthopedic trauma [7]. Most patients with orthopedic trauma have open wounds, and the fracture area is damaged, resulting in their connection with the outside world. The external environment, such as hospitals and outdoors, has many risk factors, which can easily lead to adverse reactions in patients with orthopedic trauma [8]. Wound infection is a complication that often occurs in patients with orthopedic trauma, which aggravates the pain of patients, reduces the quality of life of patients, prolongs the recovery time of patients, and has a negative impact on the health and safety of patients. Therefore, it is very important to prevent wound infection in patients with orthopedic trauma. This study observed the expression changes of inflammatory factors and T cell lymphocyte sets in patients with postoperative infection and collected other clinical data of patients to further analyze whether there are other clinical factors that can lead to the occurrence of postoperative infection. This paper provides theoretical guidance for timely detection and reduction of postoperative infection.

RETRACTED

The results of Elisa showed that the levels of IL-6, IL-2, and CRP in the infected group were significantly higher than those in the noninfected group. The analysis showed that IL-6, as a kind of interleukin, played a biological role as the main proinflammatory cytokine and anti-inflammatory myosin in the human body. At the same time, it also has a variety of functions in regulating inflammatory response in the human brain. For example, IL-6 is an important medium of fever and acute phase reaction, can cross the blood-brain barrier, and start to synthesize PGE2 in the hypothalamus, thus changing the temperature set point of the body [9–11]. Therefore, when the level of IL-6 is specifically upregulated, it indicates that the physiological balance of the body is destroyed and peripheral inflammatory reaction occurs. Il-2 is a member of the interleukin family. It is composed of many cells and cytokines and has a polytropic effect, which can activate T cells and promote the production of cytokines. The reason for the sharp rise of IL-2 in the serum of patients with orthopedic trauma and postoperative infection may be related to the fact that the immune system of infected patients is activated after the pathogen secretes a large number of cytokines, leading to a sustained and robust cellular and immune response. [12, 13]. In addition, CRP was also specifically expressed in the infection group, and the reason may be related to the fact that CRP is an acute reactive protein. The detectable level of CRP in the serum is low in the normal body environment, but when the body has inflammatory response, it can cause a sharp increase in a short time. This conclusion was also confirmed in this study [14, 15].

The expression rates of CD3 and CD4/CD8 in infected patients were significantly lower than those in noninfected patients, which indicated that cellular immunity, as an immune response mainly mediated by T lymphocytes, has a variety of biological functions in the body and is divided into different T lymphocyte subsets according to their functions. Among them, the level of CD3 can represent the overall cellular immune status. Therefore, when infection occurs, it indicates that the cellular immunity of human body cannot effectively eliminate the invasion of foreign microorganisms, indicating that the overall cellular immune status is poor, so the detected expression rate of CD3 is relatively low [16]. As the main immune response cell, CD4 can assist the body in antitumor immunity to a certain extent [17]. As suppressor T cells, CD8 has the ability to inhibit CD4 and B cells, and at the same time inhibits cellular immune response to a certain extent. The decreased expression of CD4/CD8 indicates the overall imbalance of the immune environment of the body and the low function of immune cells, so postoperative infection is more likely to occur [18]. Based on the specific expression of IL-6, IL-2, CRP and CD3, and CD4/CD8 in the T cell lymphocyte population, this study observed the efficacy of their combined detection in the evaluation of postoperative infection by drawing the ROC curve. The results showed that single indicator detection also had a certain efficacy in the evaluation of postoperative infection. However, the sensitivity and specificity of combined detection are higher than those of any single detection, and the diagnostic efficiency is higher. It is suggested that venous blood should be taken immediately after surgery and the above related indicators should be analyzed, and the corresponding postoperative antibiotic treatment should be performed according to the detection to further reduce the occurrence of infection.

RETRACTED

In addition, the other clinical data of patients also showed that the operation time, the number of combined underlying diseases, and surgical methods were the risk factors of postoperative infection in orthopedic trauma patients. The longer the operation time means that the patient's wound is exposed to the air for a longer time, and the more external bacteria and microorganisms invade, so postoperative infection is more likely to occur [19]. However, the excessive number of combined underlying diseases indicates that the patient's own internal environment is disorganized and the anti-infection ability is low, so the body's immune system is not sensitive to external microbial invasion, and it is more likely to cause postoperative infection [20]. Compared with patients undergoing elective surgery, emergency patients do not have enough time to prepare for preoperative disinfection and are rushed to clean the wound, so the number of pathogen invasion will be significantly higher than that of patients with surgical preparation, so the postoperative infection rate will increase [21].

## 3. Clinical Information and the Proposed Treatment Methods

### 3.1. Clinical Information

From January 2020 to January 2022, 98 hospitalized patients with infection and 98 patients without infection in orthopedics department during the same period are selected as the research objects. The clinical information of the subjects is collected by the clinical information questionnaire, including age, gender, BMI, history of underlying diseases, operation time, and intraoperative blood loss. All patients obtained the right to know and consent for this study and allowed to collect the clinical data for correlation analysis. Patients with congenital immune dysfunction, other malignant tumors, and poor treatment compliance are excluded.

RETRACTED

### 3.2. The Proposed Treatment Methods

#### 3.2.1. Detection of Inflammatory Factors

The serum levels of IL-6, TNF-*α*, CRP, and IL-2 are detected by ELISA. The venous blood of patients in each group is collected and put into a centrifuge after anticoagulant treatment. The centrifugation parameters are set at 3000 rpm, 12.5 cm, and 10 min. The antigen diluted with the coated liquid is carefully absorbed with a 0.2 ml straw covered with a rubber suction head, and 0.1 ml is accurately dripped into each plastic plate hole along the hole wall to prevent bubbles. The antigen is left overnight at 37°C. Quickly shake the plastic plate and pour out the coating liquid. Use another straw to absorb the washing liquid, add into the plate hole, the amount of washing liquid to fill should not overflow the plate hole, incubate 3 minutes at room temperature, throw out the washing liquid, then add the washing liquid, and repeat the above operation three times. With three 0.2 ml straws covered with rubber suction head, carefully absorb the diluted blood (to be tested, positive, and negative serum), accurately add 0.1 ml into the corresponding plate well, add 0.1 ml washing solution to the fourth well, place the serum at 37°C for 10 minutes, and then throw out the washing solution three times. Use the straw to carefully and accurately add 0.1 mL enzyme-labeled antibody along the upper part of the hole wall (do not stain the straw with serum), place it at 37°C for 10 minutes, same as above, empty, and wash three times; H_2_O_2_ is added to the substrate solution according to the proportion, and the solution is immediately absorbed with a straw, and then added to the plate well, 0.1 ml per well, and placed at 37°C for 5-15 min. After the positive control has obvious color, a drop of 2 mol/L H_2_SO_4_ is added immediately to terminate the reaction, and the OD value is measured by using a microplate reader. The kits for IL-6, TNF-*α*, CRP, and IL-2 are provided by Shanghai Enzyme-linked Biotechnology, and the item numbers are ML081887, ML081627, ML063813, and ML096281, respectively.

#### 3.2.2. Detection of T Cell Lymphoid Population

Fasting peripheral venous blood is collected from each group (avoid the central venous catheterization site). The levels of CD3, CD4, and CD4/CD8 cells in peripheral blood are detected by EP-ICS-XL flow cytometry (Beckman Coulter Co, USA) and three-color flow cytometry.

RETRACTED

### 3.3. Statistical Methods

SPSS 25.0 statistical software is used for data analysis. Measurement data are as follows: if the data obeyed normal distribution and homogeneity of variance after normality test, it is expressed as mean ± standard deviation, and paired sample *t*-test is used within the group. Enumeration data are as follows: descriptive statistical analysis is performed by percentage, and *x*^2^ test is used. Receiver Operating Characteristic (ROC) curve is used to analyze the diagnostic value. Binary logistic analysis is used to analyze the risk factors. *P* < 0.05 is considered a significant difference.

## 4. Experimental Results

### 4.1. Comparison of Baseline Data of Patients between the Infection Group and Noninfection Group

Table 1 shows the comparison of baseline data. It can be seen from Table 1 that there is no difference in postoperative infection caused by age, gender, BMI, etc., which is comparable between the two groups.

### 4.2. Comparison of Inflammatory Factors between the Infection Group and Noninfection Group

Table 2 shows the differences in inflammatory factors between the two groups. It can be seen from Table 2 that there are significant differences in the expression of IL-6, IL-2, and CRP in the inflammatory factors between the two groups.  Figure 1 shows the quantile diagram of the expression of inflammatory factors in the two groups.  Figure 1 can more intuitively observe the expression distribution of each inflammatory factor in the two groups.

### 4.3. Differences of T Cell Lymphocyte Sets between the Infected Group and the Noninfected Group

Table 3 shows the comparison of T cell lymphocyte levels between the infected group and the noninfected group. It can be seen from Table 3 that the CD3 and CD4/CD8 ratio in the infected group is significantly lower than those in the noninfected group. Although the CD4 expression rate is also decreased, there is no significant difference between the two groups.

### 4.4. Diagnostic Efficacy of Inflammatory Factors and T Lymphocyte Sets in Postoperative Infection of Orthopedic Trauma Patients

Table 4 shows the diagnostic efficiency of each index.  Figure 2 shows the diagnostic curves of each index. It can be seen from the above experimental results that IL-6, IL-2, and CRP combined with CD3 and CD4/CD8 have a high diagnostic efficiency in the diagnosis of postoperative infection. The patient's peripheral blood can be taken to detect the above indicators in time after surgery to effectively evaluate whether postoperative infection occurs.

### 4.5. Comparison of Clinical Data between the Infection Group and the Noninfection Group

Table 5 shows the comparison of clinical data. It can be seen from Table 5 that there are significant differences in the clinical data between the two groups in operation time, number of underlying diseases, and surgical methods.

RETRACTED

### 4.6. Logistic Regression Model Analysis of the Influencing Factors of Postoperative Infection in Patients with Orthopedic Trauma

Table 6 shows the logistic regression model analysis of risk factors for postoperative infection in patients with orthopedic trauma.  Figure 3 shows the multiple regression forest map. It can be seen from Table 6 and Figure 3 that IL-6, IL-2, CRP, CD3, CD4/CD8, operation time, number of combined underlying diseases, and surgical methods are risk factors for postoperative infection in patients with orthopedic trauma.

## 5. Conclusion

A retrospective study is conducted on orthopedic trauma patients in our hospital from January 2020 to January 2022. Increased inflammatory factors, T cell lymphoid disorder, longer operation time, more underlying diseases, and emergency treatment are risk factors for postoperative infection in patients with infection. Therefore, reasonable control of operation time, immediate postoperative detection of inflammatory factors, and T cell lymphocyte sets in patients with underlying diseases and emergency are of great clinical significance for early detection of infection probability, timely intervention, and reduction of infection incidence.

## Figures and Tables

**Figure 1:** Quantile diagram of the expression of inflammatory factors in the two groups: (a) the expression of IL-6 in the two groups; (b) the expression of IL-2 in the two groups; (c) the expression of CRP in the two groups; and (d) the expression of TNF-*α* in the two groups.

**Figure 2:** Diagnostic curves of each index.

**Figure 3:** Multiple regression forest map.

**Table 1:** Comparison of baseline data.

Group	*n*	Age (years)	Gender		BMI (kg/m^2^)
			Men	Women	
Infection group	98	41.84 ± 12.07	51 (52.04)	47 (47.96)	24.85 ± 1.20
Uninfected group	98	43.06 ± 11.95	55 (56.12)	44 (43.88)	25.06 ± 1.11
*t*/*x*^2^		−0.714	0.329		−1.239
*P*		0.476	0.566		0.217

**Table 2:** Differences in inflammatory factors between the two groups.

Group	*n*	IL-6 (ng/L)	IL-2 (pg/ml)	CRP (mg/L)	TNF-*α* (ng/L)
Infection group	98	40.53 ± 6.75	226.07 ± 14.62	37.46 ± 4.01	2.85 ± 0.21
Uninfected group	98	13.80 ± 1.99	131.27 ± 19.34	17.43 ± 2.42	2.81 ± 0.23
*t*		37.609	38.713	42.307	1.266
*P*		<0.001	<0.001	<0.001	0.207

**Table 3:** Comparison of T cell lymphocyte levels between the infected group and the noninfected group.

Group	*n*	CD3 (%)	CD4 (%)	CD4/CD8 (%)
Infection group	98	59.18 ± 5.51	35.94 ± 3.37	0.90 ± 0.06
Uninfected group	98	65.01 ± 5.79	36.01 ± 3.46	1.22 ± 1.24
*T*		−7.218	0.396	−22.441
*P*		<0.001	0.693	<0.001

RETRACTED

**Table 4:** Diagnostic efficiency of each index.

	95% CI	Sensitivity (%)	Specificity (%)	AUC	Cutoff value
Joint detection	0.829∼0.928	88.70	84.40	0.878	—
IL-6	0.634∼0.775	72.30	71.20	0.704	31.29 ng/L
IL-2	0.602∼0.746	68.80	61.30	0.674	182.49pg/ml
CRP	0.580∼0.730	64.50	62.20	0.655	23.64 mg/L
CD3	0.513∼0.665	66.50	62.50	0.589	61.24%
CD4/CD8	0.585∼0.733	64.30	59.30	0.659	1.02%

**Table 5:** Comparison of clinical data.

	Infection group (*n* = 98)	Uninfected group (*n* = 98)	*t*/*x*^2^	*P*
Operating time (h)	2.04 ± 0.35	1.52 ± 0.21	12.760	<0.001
Bleeding (ml)	988.65 ± 186.05	974.16 ± 181.24	0.552	0.581

Number of combined underlying diseases			32.113	<0.001
1	11 (11.22)	28 (28.57)		
2∼3	38 (38.78)	57 (58.16)		
>3	49 (50.00)	13 (13.27)		

Operation method			12.864	<0.001
Emergency department	66 (67.35)	41 (41.84)		
Select a date	32 (32.65)	57 (58.16)		

Volume of drainage (ml)			0.223	0.637
<1000	87 (88.78)	89 (90.82)		
≥1000	11 (11.22)	9 (9.18)		

Smoking			0.329	0.566
Y	55 (56.12)	51 (52.04)		
N	43 (43.88)	47 (47.96)		

**Table 6:** Logistic regression model analysis of risk factors for postoperative infection in patients with orthopedic trauma.

Risk factor	B	S.E.	Wald	P	OR	95% CI
IL-6	1.119	1.183	4.852	0.002	0.184	0.087∼0.683
IL-2	1.139	1.248	7.371	0.011	0.274	0.021∼0.592
CRP	1.472	0.741	5.271	0.017	0.462	0.281∼0.673
CD3	3.283	1.246	3.842	0.021	0.631	0.183∼0.895
CD4/CD8	1.872	1.283	6.384	0.003	0.261	0.018∼0.563
Operating time	1.629	0.982	4.371	0.019	0.173	0.076∼0.735
Number of combined underlying diseases	2.342	1.273	3.285	0.008	0.318	0.173∼0.872
Operation method	3.192	2.371	7.542	0.010	0.472	0.271∼0.816

## Data Availability

The simulation experiment data used to support the findings of this study are available from the corresponding author upon request.
